# Evidence for an African Cluster of Human Head and Body Lice with Variable Colors and Interbreeding of Lice between Continents

This article has been retracted.

**DOI:** 10.1371/journal.pone.0037804

**Published:** 2012-05-25

**Authors:** Aurélie Veracx, Amina Boutellis, Vicky Merhej, Georges Diatta, Didier Raoult

**Affiliations:** 1 Unité de Recherche sur les Maladies Infectieuses et Tropicales Emergentes, UMR CNRS 6236, IRD 198, IFR48, Faculté de Médecine, Université de la Méditerranée, Marseille, France; 2 Institut de Recherche pour le Développement, Campus International de Recherche IRD/UCAD, Hann, UMR 198 URMITE, Dakar, Senegal; Biomedical Research Institute, United States of America

## Abstract

**Background:**

Human head lice and body lice have been classified based on phenotypic characteristics, including geographical source, ecotype (preferred egg laying site hair or clothes), shape and color. More recently, genotypic studies have been based on mitochondrial genes, nuclear genes and intergenic spacers. Mitochondrial genetic analysis reclassified lice into three genotypes (A, B and C). However, no previous study has attempted to correlate both genotypic and phenotypic data.

**Materials and Methods:**

Lice were collected in four African countries: Senegal, Burundi, Rwanda and Ethiopia and were photographed to compare their colors. The Multi-Spacer-Typing (MST) method was used to genotype lice belonging to the worldwide Clade A, allowing a comparison of phenotypic and genotypic data.

**Results:**

No congruence between louse color and genotype has been identified. Phylogenetic analysis of the spacer PM2, performed including lice from other sources, showed the existence of an African cluster of human lice. However, the analysis of other spacers suggested that lice from different areas are interbreeding.

**Conclusions:**

We identified two geotypes of Clade A head and body lice including one that is specifically African, that can be either black or grey and can live on the head or in clothing. We also hypothesized that lice from different areas are interbreeding.

## Introduction

Humans are infested by two genera of lice: *Pthirus* and *Pediculus*. The *Pediculus* genus has been studied for decades and is classified based on its ecology, shape and color [1]–[14]. Two ecological forms of *Pediculus* lice may be distinguished: head lice and body lice. The head louse, *Pediculus humanus capitis*, lives and lays its eggs on hairs, whereas the body louse, *Pediculus humanus humanus*, lives and lays its eggs in clothing [7]. Differences in shape between head and body lice have also been described, but these criteria have not been shown to be relevant enough to divide the two into distinct species [12]. Also, louse coloration was described in the beginning of the 20^th^ century, and it was noted that lice have different colors depending on their geographic region and the color of their host's skin [3], [8], [9], [11]. A series of gradations between the black head or body louse of West Africa and the light dirty grey head or body louse of Europe was described [10], [13], [14].

Later, researchers began performing genetic studies on lice [15]–[23]. First, a study based on the 18S ribosomal RNA gene reported that head and body lice were not phylogenetically distinct. In fact, two phylogenetic groups were described: the Sub-Saharan African lice and other lice that are distributed elsewhere worldwide. Each of these groups contained two distinct subgroups: head and body lice [23]. The divergence of human head and body lice was considered to be a recent event occurring within each of the geographical groups. A second phylogenetic study was based on mitochondrial genes [21], [22]. This allowed the description of three phylogenetically different clades of lice: the “most common worldwide clade”, which comprises both head and body lice (called Clade A), the “head lice only clade”, found in America, Europe and Australia (called Clade B), and “another head lice only clade”, which was first found in Nepal and Ethiopia [21] but was also recently found in Senegal [24] (called Clade C). Finally, another phylogenetic study of Clade A lice based on intergenic spacers (Multi-Spacer-Typing method or MST) reported two clusters of lice: Non-African lice (which we will call A1) and African lice (which we will call A2) [20].

Since then, there have been no studies aiming to correlate phenotype and genotype in human lice. Therefore, we wanted to examine both aspects to determine whether there is any correlation among the color, geographical source, ecotype (head and body) and phylogeny of lice. For this approach, we used Clade A lice collected in Senegal, Burundi, Rwanda and Ethiopia. They were photographed and then genotyped with the MST method [20]. To complete the phylogenetic analysis of our data, we also used previously genotyped Clade A lice from African and Non-African regions [20].

## Materials and Methods

### Ethics statement

Informed verbal consents were obtained from all the participants involved in our study. All participants of this study were illiterate. It is why a verbal informed consent procedure was preferred over written consent. The Ethic Committee of the Institute Fédératif de Recherche approves this verbal consent procedure as it is in accordance with the French Bioethics law N° 2004-800 60 (06/08/2004). Dr Oleg Mediannikov participated in the collection and was a witness of the participant's consents. Local authorities (village chief) approved, and were also present. This study was approved (Agreement #12-004), by the Ethic Committee of the Institute Fédératif de Recherche 48, Marseilles, France since this study was a non-interventional epidemiological research study as a part of the French Bioethics law N° 2004-800 (06/08/2004). The poorest districts of Dakar were chosen because of the highest possibility to find lice. Girls are more likely to have long hairs (boys are often shaved). Lice were anonymized before processing for genetic analysis.

### The study

In this study, we had four parameters to compare: ecology, geographical origin, phylogeny based on 4 spacers and color. So we decided to sequence only Clade A lice because this is the only clade that comprise both head and body lice and therefore is a specific problem of public health as body lice are vectors of outbreaks. Lice from four countries were genotyped with the MST method including head lice from Senegal collected in October and November 2010 [24], body lice from Southern Ethiopia collected in 2010 [25], body lice from Rwanda collected in 2011 (three lice per individual) and both head and body lice from Burundi collected in 2008 (three lice of each ecotype per individual). Altogether, 19 Clade A lice were used in this study (Table 1). All lice were stored at −20°C before DNA extraction with the QiAamp Tissue kit (QIAGEN, Hilden, Germany). Senegalese and Rwandan lice were photographed with a camera (Olympus DP71) fixed on a low power stereo microscope (Olympus SZX16). The lice from Ethiopia and France were photographed in the field (with a Nikon D90) either in the hand of one of the authors (Ethiopia) or directly on the clothes of the infested person (France). Four intergenic spacers (S2, S5, PM1, PM2) known to be very polymorphic [20] were used in this study. The sequencing was performed following the protocol previously described [20] with some minor modifications. Briefly, the PCR reactions were prepared on ice and contained 3 µl of the DNA template, 4 µl of Phusion HF Buffer, 250 µM of each nucleotide, 0.5 µM of each primer, 0.2 µl of Phusion DNA Polymerase (Ozyme) and water to a final reaction mixture volume of 20 µl. The reactions were performed in a PTC-200 automated thermal cycler (MJ research, Waltham, MA, USA). The cycling conditions were 98°C for 30 sec; 35 cycles of 5 sec at 98°C, 30 sec at 56°C, 15 sec at 72°C; and a final extension time of 5 min at 72°C. The success of the PCR amplification was then verified by migration of the PCR product on an agarose gel. The NucleoFast 96 PCR Plates (Macherey-Nagel EURL, France) and BigDye Terminator version 1.1 cycle sequencing-ready reaction mix (Applied Biosystems, Foster City, CA) were then used to purify the PCR products before sequencing in both directions with the same primers used in the PCR amplification. The ABI 3100 automated sequencer (Applied Biosystems) resolved the sequenced products. The program ChromasPro was used to analyze, assemble and correct the sequences. When forward and reverse sequences could not be assembled, they were analyzed separately and resolved. Each sequence was aligned with genotypes published in Genbank [20]) for identification. When less than 100% homology was obtained, the new genotype was recorded, a new number was assigned to it and sequences were deposited in Genbank under accession numbers from JQ652371 and JQ652455. When the chromatogram indicated possible heterozygotic sequences, these samples were cloned to identify the different allelic sequences. The PCR products were cloned into pGEM-T-Easy vector (Promega, Madison, WI) following the manufacturer's instructions with some minor modifications. Before ligation, A-overhangs were added to the PCR product. This was performed by incubating 4.2 µl of purified PCR product with 1 U of DyNAzyme II DNA polymerase, 0.5 µl of Optimized DyNAzyme Buffer and 0.2 mM dATP with a final volume of 5 µl for 20 min at 72°C. Then, each reaction was ligated with 5 µl of 2X Rapid Ligation Buffer, 3 µl of purified A-overhangs-PCR product, 1 µl of T4 DNA ligase and 1 µl of pGEM®-T Easy Vector and incubated overnight at 15°C. Each ligation reaction was transformed into 50 µl of JM109 High Efficiency Competent Cells by letting them incubate together on ice for 20 min before a 1 min heat shock in a 42°C water bath. 950 µl of LB broth was then added to cells before incubation on a 37°C shaker for 1.5 hours. 300 µl of transformed cells was plated onto LBagar/ampicillin/IPTG/X-Gal plates and these were incubated overnight at 37°C. Eight white colonies per sample were then resuspended in 100 µl of RNase/DNase free water and subsequently PCR amplified and sequenced using the M13 universal and M13 reverse primers. Phylogenetic analysis was done using our data and data from a previous study performed in 2010, which included lice from France, Portugal, Mexico, Russia, Burundi and Rwanda (these lice were given names beginning with “li-” in the trees) [20]. Two phylogenetic methods, Maximum Parsimony (MP) and Maximum Likelihood (ML), were used to infer the trees for each individual spacer. For each spacer, the louse nucleic sequences were aligned with the genotype 1 found in Genbank (EU928781.1, EU928804.1, EU913096.1, EU913178.1 for PM1, PM2, S2 and S5, respectively) using the MUSCLE algorithm [26]. Then, trees were drawn within the MEGA 5 software with complete deletion [27]. A tree was also constructed with the concatenated sequences of the four spacers (S2, S5, PM1, PM2). Because the louse genome is diploid, in instances where there were two different alleles per locus, all possibilities of concatenation were made for each louse and all of them were taken into account in the tree (the possibilities were labeled from a to h in the tree).

**Table 1:** Results of the Multi-Spacer-Typing of African lice.

Country	Type	Host ID	Louse ID	Spacer S2	Spacer S5	Spacer PM1	Spacer PM2
Senegal 2010	HEAD	1	12	**83**	36/42	13	**60/61**
			13	**83/84**	42	13	**60/62**
		2	14	NA	36/42	13	NA
		3	48	**85/86**	8/36	13	**63/64**
		4	94	**87**	8	13	**65/66**
			95	**87**	8/42	13	**66**
		5	181	**89**	**47**	13	43
		6	214	NA	35	13	**65**
		7	223	**90**	8/36	13	**67**
		8	226	**91/92**	**36/62**	13	**62/68**
Ethiopia 2010	BODY	9	2408	**100**	36	4/5	**85/87**
		10	2409	**96**	**54/59**	18	**83/92**
Burundi 2008	HEAD	11	2394	**97/101**	**35/53**	**25/34**	**82**
		12	2395	**93**	**51**	**35**	**76**
	BODY	13	2396	76	35	17	**80/74**
		14	2397	76	32/36	17	**69**
Rwanda 2011	BODY	15	2400	**103**	**36/54**	4	**69/70**
		16	2401	**108**	**50**	4	**92**
		17	2402	**104**	**60**	3/4	**86**

In case of heterozygocy, the numbers of the two genotypes were mentioned.

NA, not available.

New genotypes in bold.

## Results

Clade A lice collected from Senegal, Burundi and Rwanda (head or body) were all black. Clade A body lice collected in southern Ethiopia and lice collected in France were grey (Figure 1). Head lice collected in Ethiopia were black, belonged to genotype C and were not included here [25]. Photographs of genotyped lice from other Non-African regions (Russia, Portugal, Mexico) and from Burundi were not available. After sequencing (Table 1), many new genotypes were found, especially for S2 and PM2 spacers, but there were also new genotypes for spacers S5 and PM1. In Senegal, all 10 tested lice had genotype 13 for spacer PM1. The other spacers had higher variation. We found that some lice collected from the same human host have the same genotype (lice 12 and 13 and lice 94 and 95). There is a lack of data for lice 14 and 214 due to the failure of spacer S2 to amplify, despite three attempts and a good positive control. Moreover, for spacer PM2 of louse 14, the amplification was non-specific on three attempts.

**Figure 1:** Pictures of lice.

Phylogenetic analysis was performed including lice from other sources [20], and trees were drawn for each of the four spacers. Altogether, 55 Non-African lice and 40 African lice were included in the analysis. The same tree topologies were found with Maximum Likelihood (ML) and Maximum Parsimony (MP) methods. However, the topologies of the trees constructed with the different spacers were not congruent and had low bootstrap support (Figures 2B and 3). The tree from spacer PM2 showed two distinct clusters: African lice separated from Non-African lice, which was supported by a 54% bootstrap (Figure 2B). The analysis of the sequence alignment of the spacer PM2 showed two positions at which single-base substitutions allowed us to distinguish African lice from lice coming from other regions: positions 26 (T in Africa and A out of Africa) and 31 (A or C in Africa and T out of Africa) and may have caused the observed clustering (Figure 2A). The only exception is the Senegalese louse 181 that clustered with Non-African lice in the tree (Figure 2B) and has the same signature than Non-African lice have at these positions (not shown). For spacers PM1, S2 and S5, no such clustering was observed (Figure 3, A to C). When concatenated sequences of the four intergenic spacers were used (Figure 3D), the resulting tree had the same topology as the PM2 spacer tree, but with a 43% bootstrap. Given that phylogenetic analysis of spacer PM2 sequences showed a correlation between geography and genotype, the proportion of each genotype found in African and/or Non-African countries (Geotyping) was compared for each spacer (Figure 4). We represented in the circles only genotypes found in two or more lice; the others genotypes were grouped and called “others.” Spacers PM2 and S2 (67 and 55 different genotypes) were more variable than PM1 and S5 (25 and 34 different genotypes). In several cases, genotypes were shared between African and Non-African lice in each spacer. However, in the PM2 spacer, this was very rare, as only one louse from Senegal (louse 181) and one louse from Russia had the same genotype (genotype 43). All other genotypes were not shared by African and Non-African countries. In spacer S5, two genotypes were shared between the two geographic areas: genotype 8 (Senegal and Moscow) and 42 (Senegal, Rwanda, France, Mexico and Moscow). In spacer S2, one genotype was shared: genotype 39 (Burundi and Mexico). However, it was in spacer PM1 that the biggest proportion of lice were observed to have genotypes shared by the two areas. Indeed, genotypes 13 and 18 were the most prevalent genotypes (respectively 30 and 33% of genotyped lice) and were found both in African and non-African countries: genotype 13 was found in Senegal, France and Portugal and genotype 18 was found in Rwanda, Ethiopia, Mexico and Russia (Figure 5).

**Figure 2:** Spacer PM2 analysis. Phylogenetic analysis of African (black) and Non African lice (blue) (A) The first 69 bp of the alignment of a subset of PM2 spacer sequences. Two polymorphisms (shown with arrows) discriminate between African and Non-African lice (B) Phylogenetic tree based on PM2 sequences using Maximum likelihood method. For lice being heterozygote in PM2 spacer, the two alleles were included in the tree and they were called the same with one letter “a” or “b” to distinct them.

**Figure 3:** Analysis of spacer PM1, S2, S5 and concatenation of the four spacers. Phylogenetic analysis of African (black) and Non African lice (blue) using Maximum likelihood method based on spacer PM1 (A), spacer S2 (B), spacer S5 (C), the concatenation of the four spacers (D). For lice being heterozygote, the two alleles were included in the trees and they were called the same with one letter “a” or “b” to distinct them.

**Figure 4:** Proportion of each genotype among African (black) and Non-African (blue) lice. The name (ID numbers) of the genotypes found in both African and Non African countries were framed. Genotypes (either African and Non African) found in only one louse were not represented and were grouped as “others”.

**Figure 5:** Geographic repartition of the four spacers genotypes. Genotypes found in at least two countries are colored (one color per genotype) and genotypes found in only one country are in white. The size of the symbols vary with the number of lice found for each genotype. Only genotypes found in at least two lice were represented.

Altogether, these data show a correlation between geography and genotype but only in spacer PM2. Moreover, among the four spacers studied, none showed a correlation between the ecotype and the genotype, as head and body lice were not separated in the phylogenetic trees. Finally, no correlation has been observed between louse color and genotype as we did not find black and grey lice separately clustered in the trees.

## Discussion

In this study, MST based on the four intergenic spacers S2, S5, PM1 and PM2 was confirmed to be a very sensitive method that is able to discriminate among individuals. The observation of identical genotypes from the sequences of two lice collected on the same person strengthens our faith in the reliability of the method. This method therefore appears to be well adapted for the study of human lice and able to address population-level questions.

Our first observation was that the PM1 genotype 13 appeared in all Senegalese lice, but not in lice from Burundi, Rwanda and Ethiopia. This genotype was also found in lice from France and Portugal [20]. This observation that lice from Senegal and France have the same genotype on spacer PM1 suggested that interbreeding has occurred between lice from these two countries. As the French have been in Senegal since the XVIII century, this hypothesis is historically logical. Genotype 18 is also prevalent in African and Non-African countries (Figure 4), supporting the possibility that lice from different continents are interbreeding.

When the frequency of the genotypes of the PM2 spacer were observed, it was noted that this spacer was the most variable among those tested and that only one louse from Senegal had the same genotype as a louse from Russia. In all other cases, African and Non-African lice harbored distinct genotypes, as confirmed by the phylogenetic tree that showed a cluster of African lice (54% extra support), regardless of the method used. This topology was similar to that of a previous study based on 18S rRNA [23]. However, with the MST method, head and body lice did not cluster separately inside their geographic cluster, as opposed to the results observed when using 18S-based phylogeny. Finally, when concatenated sequences of the four spacers were used, the resulting tree conserved the same topology as the PM2 tree but with lower bootstrap values. This showed the importance of first drawing separated trees for each spacer before drawing concatenated trees when using the MST method. This allows researchers to check if the different spacers tell the same story.

In conclusion, a clear correlation between genotype and phenotype could not be shown. First, a correlation between genotype and geographic origin was observed, but only with spacer PM2. Second, there was no correlation between color and genotype or ecotype (head and body). Moreover, contrary to results from previous studies [3], [8], [9], [11], the color of lice may not be linked to the color of the host's skin as grey body lice were found on black hosts in Ethiopia.
